The article "Divergent Analyses of Genetic Relatedness and Evidence-Based Assessment of Therapeutics of Staphylococcus aureus from Semi-intensive Dairy Systems" was retracted in 2024. Reasons: signs of a paper mill; suspected computer-generated content; unreliable results or conclusions; concerns about the data.

# Divergent Analyses of Genetic Relatedness and Evidence-Based Assessment of Therapeutics of *Staphylococcus aureus* from Semi-intensive Dairy Systems

**DOI:** 10.1155/2022/5313654

**Published:** 2022-06-20

**Authors:** Sidra Aziz, Nahla Muhammad Saeed, Hiewa Othman Dyary, Muhammad Muddassir Ali, Rao Zahid Abbas, Aziz ur Rehman, Sammina Mahmood, Laiba Shafique, Zaeem Sarwar, Fakhara Khanum, Tean Zaheer, Khurram Ashfaq, Mughees Aizaz Alvi, Muhammad Shafeeq, Arslan Saleem, Amjad Islam Aqib

**Affiliations:** ^1^Tehsil Headquarter Hospital, Mankera, Pakistan; ^2^College of Veterinary Medicine, University of Sulaimani, Sulaymaniyah, Kurdistan Region, Iraq; ^3^Institute of Biochemistry and Biotechnology, University of Veterinary and Animal Sciences, Lahore 54000, Pakistan; ^4^Department of Parasitology, University of Agriculture, Faisalabad 38000, Pakistan; ^5^Department of Pathobiology, University of Veterinary and Animal Sciences, Lahore Sub-Campus, Jhang 35200, Pakistan; ^6^Department of Botany, Division of Science and Technology, University of Education, Lahore 54000, Pakistan; ^7^State Key Laboratory for Conservation and Utilization of Subtropical Agro-Bioresources, Guangxi University, Nanning 530005, China; ^8^Department of Theriogenology, Cholistan University of Veterinary and Animal Sciences, Bahawalpur 63100, Pakistan; ^9^Department of Food Science and Technology, Government College Women University, Faisalabad 38000, Pakistan; ^10^Department of Clinical Medicine and Surgery, University of Agriculture, Faisalabad 38000, Pakistan; ^11^Department of Aerospace and Geodesy, Technical University of Munich Arcisstr. 21, 80333 Munich, Germany; ^12^Department of Medicine, Cholistan University of Veterinary and Animal Sciences, Bahawalpur 63100, Pakistan

## Abstract

Use of antibiotics without following standard guidelines is routine practice in developing countries which is giving rise to genetic divergence and increased drug resistance. The current study analyzed genetic divergence and drug resistance by *S. aureus* and therapeutic efficacy of novel antibiotic combinations. The study revealed that 42.30% (minimum 20%-maximum 70%) of milk samples are positive for *S. aureus*. Study also revealed seven SNPs in the *S. aureus nuc* gene (c.53A>G, c.61A>G, c.73T>C, c.93C>A, c.217C>T, c.280T>C, and c.331T>A). Local isolates Staph-2 and Staph-3 were closely related to *Bos taurus nuc* gene (bovine *S. aureus*), while Staph-1 was closely related to *Homo sapiens* (human *S. aureus*) indicating shifting of host. Change of two amino acids and staphylococcal nuclease conserved domain was observed in all local isolates of *S. aureus*. The isoelectric points predicted by protParam of Staph-1, Staph-2, and Staph-3 proteins were 9.30, 9.20, and 9.20, respectively. The antibiotic susceptibility profile of *S. aureus* presented highest resistance against penicillin (46.67%) and glycopeptide (43.33%). When a single antibiotic regimen was adopted in a field trial, the highest efficacy was reported in the case of oxytetracycline (80%) while lowest was presented by azithromycin. Among antibiotics' combined regimen, the highest efficacy (80%) was presented by gentamicin with oxytetracycline: cefotaxime with vancomycin; and ciprofloxacin with vancomycin. The current study concluded rising percentages of *S. aureus* from dairy milk, proofs of genetic host shifts, and altered responses of in on field therapeutics.

## 1. Introduction

Semi-intensive dairy systems represent 21% of milk production in Mexican dairy milk collection systems [1], while in other parts of the world, predominantly Asian countries, it is increasing day by day. Losses are attributed to the spread of different bacteria salient of which is *Staphylococcus aureus* (*S. aureus*). This bacterium is commensal and opportunistic that can colonize various animal species and humans [2]. The bacteria cause severe infections in humans and animals. The former infection involves skin and soft tissue infection (SSTI), which is clinically manifested as puffy infectious blood vessels, abscesses, papules, tuberculosis, and Staphylococcal scalded skin syndrome (SSSS). Isolated infections include toxic shock syndrome (TSS), pneumonia, or neonatal TSS-like human excitation [3]. Skin, mucous membrane, upper and lower respiratory tract, and urogenital tract are significant attacking sites in humans and animals [4, 5]. Pathogens may appear as fatal due to septic shock following intramammary infections in animals [6].

*S. aureus* is a widespread and infectious pathogen that exists in 30-40% of all cases of mastitis and 80% of subclinical bovine mastitis which may cost 35 USD yearly as losses worldwide [7, 8]. The capability of producing mastitis is governed by numerous virulence factors that are structural or secretory [9, 10]. The structural virulence factors belong to adhesions, protein A, and capsular polysaccharide, whereas in secretory proteases, hemolysins, coagulase, lipase, and hyaluronidase are included [11, 12]. Infection increases due to increased resistance to multiple antibiotics such as methicillin-resistant *S. aureus* (MRSA). Spread of this pathogen is restricted not only to bovine but also to other animals like goats [13]. Newer strains of *S. aureus*, i.e., vancomycin-resistant *S. aureus* (VRSA), are also rising in bovine milk [14] in addition to already reported MRSAs. These strains are the most common cause of food poisoning and hospital infections [15–17] because of exoenzymes, exoproteins, and toxins [15, 18]. Ancestry analysis provided specificity within animals that is now changed to host shifts from one animal to another. Moreover, the pathogen is required to be considered for studying phenomena of protein folding and other molecular structures [16, 19].

*S. aureus* has the ability to yield extracellular thermostable nuclease, which is encoded by *nuc gene*. Among several other genes, this gene is found successful in distinguishing *S. aureus* in staphylococcal spp. This gene is thus considered a specific marker of *S. aureus* identification through PCR [16]. There are several researchers reporting *nuc* gene as a fast and reliable identification marker for *S. aureus*. Specificity and sensitivity of *nuc* gene to identify *S. aureus* have been reported as 89.6% and 93.3%, respectively [20]. Keeping in view the influencing semi-intensive dairy systems, this study aimed at (a) probing divergence of genetic relatedness of *S. aureus* within host and across host, (b) estimating the modified pattern of drug resistance profile against all classes of antibiotics, and (c) finding response of single and double antibiotic regimens against *S. aureus*-based clinical mastitis.

## 2. Results

### 2.1. Genetic Relatedness for Host Shift Analysis

Molecular identification of biochemically characterized *S. aureus* was targeted at 500 bp of *nuc* gene. The positive samples which were made part of this genetic relatedness are also pointed out along with other positive samples in Figure 1. Alignment of nucleic acid and protein sequences is given in Figures 2 and 3, respectively. Seven SNPs were identified in the *S. aureus nuc* gene at position c.53A>G (transition), c.61A>G (transition), c.73T>C (transition), c.93C>A (transversion), c.217C>T (transition), c.280T>C (transition), and c.331T>A (transversion) (Table 1). Nucleic acid alignment revealed that Staph-1, Staph-2, and Staph-3 were 97.37%, 98.02%, and 99.13% identical with a reference sequence, respectively. A phylogenetic tree of the *S. aureus nuc* gene was constructed. Five clades were observed in the phylogenetic tree when local *S. aureus* samples were compared with the *S. aureus nuc* gene of different species (different sources) from the NCBI database. Local *S. aureus nuc* (Staph-2 and Staph-3) gene sequences were closely related to the *S. aureus nuc* isolated from *Bos taurus*. These two local isolates (Staph-2 and Staph-3) clustered together only. Staph-1 (local isolate) gene sequence was closely related to *S. aureus nuc* isolated from *Homo sapiens* (vaginal and blood). This indicated that 33.33% of host shifts as one among three isolates were related to humans. Staph-1 clustered with *Homo sapiens* (blood, stool, sputum, contaminated platelets, wound, and swab), international space station surface, pork, food, and *Bos taurus* (Figure 2). The nucleic acid motif *p* value of the reference sequence was 4.66*e* − 191. The *p* value of sample Staph-1 was 2.01*e* − 190. Staph-2 and Staph-3 have the same *p* value (1.64*e* − 191). Sequences of motifs were discriminated by different colors represented in Figure 4. The protein motif *p* value of the reference sequence was found 4.31*e* − 160 (Figure 5). The *p* value of sample Staph-1 was 1.77*e* − 159. Staph-2 and Staph-3 have the same *p* value (2.88*e* − 160). Sequences of motifs were discriminated by different colors represented in Figure 3. Nucleotide motif construction involved an 1832 bp sequence, while amino acid motif construction involved a 608 bp sequence. Frequency of adenine and thiamine nucleotide in motifs was 0.328 while cytosine and guanine frequencies were 0.172. The only coding region was involved in the nucleotide structure (Figure 6). Asparagine was replaced by aspartic acid (p.N18D), and serine was replaced by tyrosine (p.S31Y) (Table 2). The conserved domain of staphylococcal nuclease was observed in reference, Staph-1, Staph-2, and Staph-3 protein sequences. The gene structure (exonic region) of *S. aureus* nuc gene was found similar to the reference sequence (Figure 7). The protein structure of reference, Staph-1, Staph-2, and Staph-3 proteins resembles the staphylococcal nuclease protein (Figure 8). Protein-protein interaction was found in Staph-1, Staph-2, and Staph-3 proteins (Figure 9). Predicted functional partners of *S. aureus nuc* protein are given in Figure 10. STRING software predicted the association between genes based on observed patterns of simultaneous expression of genes (Figure 11).

### 2.2. Pattern of Prevalence and Drug Susceptibility Profile of *S. aureus*

The study found 42.33% (127/300) of milk samples from commercial dairy farms positive for *S. aureus*. The range of *S. aureus* prevalence at the farm level varied from 20% (three farms in the study area) to 70% (only one farm observed). Four farms presented 30-37.04%, while one farm showed a 42.8% prevalence of *S. aureus* (Figure 12). Antibiogram of *S. aureus* against 24 antibiotics from eight antibiotic groups showed varied responses. As an average effect of a class of antibiotics, penicillin and glycopeptides were found least effective in that 46.67 and 43.33% of *S. aureus* were resistant to these antibiotics (Table 3). On the other hand, fluoroquinolones, aminoglycosides, sulfonamides, macrolides, and tetracyclines were the most effective against *S. aureus* in the current study. Against cephalosporins, *S. aureus* were 36.67, 30%, and 33.33% resistant, intermediate, and sensitive, respectively. The pattern of susceptibility of isolate against individual antibiotics is shown in Figures 13(a)–13(h). There were 40-50% isolates resistant to cefoxitin, cefotaxime, sulfathiazole, oxacillin, clarithromycin, and dalbavancin. The study also showed that 60% of isolates are resistant to ampicillin and vancomycin. The highest sensitivity was found against enoxacin (80%), followed by sulfamethoxazole/trimethoprim, amikacin (70%), gentamicin (60%), azithromycin (60%), and oxytetracycline (60%). About 40% of isolates expressed intermediate susceptibility against streptomycin, cefixime, sulfaphenazole, sulfadiazine, and clarithromycin.

### 2.3. Field Trials

The study noted that oxytetracycline showed the highest efficacy (80%) among single antibiotic regimens while azithromycin showed the least efficacy (20%). Cefotaxime, vancomycin, and ciprofloxacin showed 60% efficacy while 40% of cases supported gentamicin, sulfadimidine, and azithromycin (Table 4). Combination regimens showed an 80% success rate in favor of gentamicin with oxytetracycline, cefotaxime with vancomycin, and ciprofloxacin with vancomycin. Azithromycin in combination with sulfadimidine and azithromycin with gentamicin were the least effective drug regimens found in this trial.

## 3. Discussion

The clue of host shift of *S. aureus* in the current study (one of three *S. aureus* to be closely related to humans while distantly related to cows) was in line with findings of [21]. They reported clonal complexes (CCs), i.e., CC97 *S. aureus* isolate of cattle transmitted to humans while CC22 of humans found in cattle in Algeria. Human-associated strains of *S. aureus*, e.g., CC22 MRSA which was strictly responsible for hospital-acquired MRSA and community-acquired MRSA infections [22], were reported predominantly in Germany from dogs and cats [23]. *S. aureus* genes identified in humans' milk were found in *S. aureus* isolated from bovine milk [24]. SNP identification in this study was more than those identified by [25, 26]. They found 3 SNP clades, two belonging to bovine mastitis while one clade belonging to international human isolates. SNP-based analysis indicated the combination of clades existing in humans and animals. In close agreement with the findings of the current study, 5 SNP clusters were identified in bovine mastitis [26]. In another study, 15 SNPs were identified with resembling phenotype [27]. In another study, 12 genome SNPs were identified from bovine in UK. The livestock-associated *S. aureus* strain (LA-MRSA), CC398, presented close phylogenetic relation to humans and turkeys. SNPs in the *nuc* gene lead to amino acid change revealed by in silico analysis. This change of amino acids might be associated with changes in the activity of the enzyme.

There is debate about the use of different genes to indicate differences and similarities with reported sequences. In our study, *nuc* gene was preferred for *S. aureus*. Sequence analysis and genotyping of the *S. aureus nuc* gene proved to be a suitable tool for detecting mastitis in dairy farm animals [27]. The results of [28] revealed that *nuc* genes are derived from thermophilic bacteria and picked up by common ancestor staphylococci. In a study, homology analysis revealed no significant similarities between two *nuc* genes (*nuc*1 and *nuc*2) [28]. *nuc*1 is specific to *S. aureus*. 79% identity of *nuc*2 gene was observed with *Staphylococcus epidermidis* gene. This identity suggested a close relationship of this gene with other species in the Staphylococcus genus. Phylogenetic trees of *nuc*2 and *nuc*1 genes were found in different clusters in another study [29]. Staphylococci were differentiated using the *nuc* gene similarly to 16S rRNA sequences used for taxonomy classification [20]. Homology comparison of the *nuc* gene revealed that this gene is present everywhere in the genus Staphylococcus except *Staphylococcus sciuri* [30]. More than 70% similarity with nuc2 thermonuclease protein sequence from different species of *Staphylococcus* was observed in a study. Less than 60% similarity was observed with *S. aureus* nuc1. A higher-level homology of Staphylococcus was observed in the case of *S. epidermidis* (89.3%), *Staphylococcus hominis* (84.0%), and *Staphylococcus lugdunensis* (85.6%) [28]. Other scientists also used *nuc* gene to identify *S. aureus* [31]. Hamidi and his colleagues assessed the ability of GENECUBE assays to detect *nuc* gene (identification of *S. aureus*) using a blood culture medium. They have found 100% specificity and sensitivity of GENECUBE assays in detecting *S. aureus* [32]. *S. aureus* presence in milk samples for confirmation of subclinical mastitis was examined by Hida et al. [33].

The higher prevalence of *S. aureus* contradicted with findings of another study conducted in the same country [34]. The reason for the discrepancy might be because they focused only on subclinical *S. aureus* and did not include clinical and normal milk samples. In another study, 39.03% of *S. aureus* were noted from subclinical mastitis. Another study reported a very high prevalence of *S. aureus* (61.60%) from subclinical mastitis cases [35]. Subclinical mastitis in the province of the study area revolves around 40-55%. In that context, the current study alarms to find new plans to combat this pathogen. The high rise in this pathogen is attributed to no or lack of preventive measures. The pathogen is contagious, while its transfer is reported between animal-animal, animal-human, and human-human. In a recent study, 72.91% of nasal samples produced *S. aureus*, while among these were 34.29% (24/70) pathogenic as identified by the *mecA* gene [36]. From animal sources (cat, dog, buffalo, calf, and buck), 28.7% of multiple drug-resistant *S. aureus* were noted [37]. These facts indicate the significant spread of this pathogen among dairy animals, pets, and humans.

There was 100% resistance of *S. aureus* (camel mastitis origin) against cefoxitin and oxacillin in a previous study [38]. *S. aureus* from bovine milk were found 100% sensitive to ciprofloxacin and trimethoprim/sulfamethoxazole, 90% against gentamicin and levofloxacin, 60% against tylosin, 50% against fusidic acid, and 40% against oxytetracycline [38, 39]. Another study on MRSA showed 80% sensitivity against ciprofloxacin. Resistance against antibiotics in this pathogen is attributed to extended beta-lactamase production encoded to be blaCTX-M55, ST-23 complex, ST-410, ST-167 genes, blaCTX-M15, blaCTX-M14, and ST-10. Such kind of response of antibiotics is not only confined to *S. aureus* of mastitis but also extended to *E. coli* from endometritis [40].

## 4. Materials and Methods

### 4.1. Milk Sample Collection

The study area consisted of developing commercial dairy systems with semi-intensive dairy systems in District Khanewal, Punjab, Pakistan. On a random basis, *n* = 10 dairy farms having not less than n=50 animals in milking situation but with a commercial dairy system were approached with prior consent of the farmers. A total of *n* = 300 milk samples (*n* = 30 milk samples from each farm) were collected on a convenient sampling basis. The samples were aseptically collected in sterile tubes labeled with tags and shifted to the laboratory of central diagnostic, Cholistan University of Veterinary and Animal Sciences, Bahawalpur, Pakistan.

### 4.2. Isolation and Identification of *S. aureus*

Milk samples were centrifuged at 6000 rpm/15 minutes, and the supernatant was discarded. Sterile nutrient broth was added for further incubation at 37°C for 24 hours as prescribed in previous studies [36, 37]. The incubated samples were swabbed on mannitol salt agar, and growth obtained after 24 hours at 37°C was proceeded for biochemical analysis as per guidelines of Bergey's manual of determinative bacteriology. The pooled information was used to declare confirmation of bacteria.

### 4.3. Molecular Analysis

Isolates identified from biochemical tests were put to molecular analysis. For this purpose, randomly, 50% of *S. aureus* (*n* = 64) were selected. Primers of the nuc gene were designed using Primer 3 (https://www.ncbi.nlm.nih.gov/tools/primer-blast/) software (Nuc_forward 5′AAGGGCAATACGCAAAGAG3′ and Nuc_reverse 5′AAACATAAGCAACTTTAGCCAAG3′). The reaction mixture contains PCR 2x master mix = 10 *μ*L (ThermoScientific Catalog # K0171), forward primer = 1 *μ*L (10 pmoL), reverse primer = 1 *μ*L (10 pmoL), DNA = 2 *μ*L (50 ng/L), deionized water = 6 *μ*L, and reaction volume was 20 *μ*L. Touchdown PCR (35 cycles) was used to amplify the nuc gene of *S. aureus*. Thermocycler profile includes initial denaturation 94°C (5 min), denaturation 94°C (45 sec), annealing 63°C-53°C (45 sec), extension 72°C (45 sec), and final extension 72°C (5 min). The dilutions of DNA (50 ng/*μ*L) were made, and nuc gene was amplified. After amplification, these amplicons were purified using a purification kit (Gene JET PCR Purification Kit Catalog number: K0701) and sent for sequencing. *S. aureus* positive for nuc gene and presenting multidrug resistance were sent for sequence analysis. Isolates showing similar sequences were excluded while those (*n* = 3) presenting genetic variations and showing the highest drug resistance were discussed in this paper.

Single-nucleotide polymorphisms were observed in sequencing chromatograms using chromas software. BLAST (Basic Local Alignment Search Tool) was used to check the similarity of the *S. aureus nuc* gene with the reference sequence. Clustal omega was used for the alignment of nucleic acid and protein sequences. A phylogenetic tree was constructed using Mega X. Nucleic acid and protein motifs were constructed using MEME Suit (Multiple Expectation maximizations for Motif Elicitation) [41]. The gene structure of *S. aureus nuc* gene was determined by using a gene structure display server. Swiss model software predicted the 3D structure of thermonuclease. Protein-protein interactions were determined using STRING software (Search Tool for the Retrieval of Interacting Genes/Proteins). The physical and chemical properties of proteins were predicted by protParam *S. aureus* using guidelines given in the Clinical and Laboratory Standard Institute.

### 4.4. Susceptibility Profile

The genetically identified *S. aureus* was processed to respond to eight classes of antibiotics, each with three representative antibiotics (Table 5). The Clinical and Laboratory Standard Institute's [42] instructions were used to find the susceptibility (resistant, intermediate, and sensitive) profile of bacteria by both the disc diffusion method and the broth microdilution method. Where felt necessary, European Committee on Antimicrobial Susceptibility Testing was also consulted for analysis [43]. The need for the antibiotic profile of bacteria was deemed necessary because dairy systems lack proper veterinary sanitary control and technology for milk collection. These directly affect the spread of pathogens along with their surge in resistance [44, 45].

### 4.5. Field Trial of Different Antibiotics against *S. aureus*

This trial consisted of the evaluation of different antibiotics against *S. aureus*-based clinical mastitis. The following criteria were used for this trial (Table 4, Figure 14).

#### 4.5.1. Inclusion Criteria for Antibiotics

- Field trial consisted of antibiotic groups based on their activity in *in vitro* trial
- Class of antibiotics representing more than 30% response against bacteria was included in field trial keeping in view their resistance. Penicillin was thus excluded with this criterion
- From each class, one antibiotic was selected based on its availability in the study area and its use as parenteral route to cover infection at ease
- All the antibiotics were used in a single regimen and next as a combination regimen
- Combination was made on their apparent mode of action, i.e., bacteriostatic was used in combination with bacteriostatic while bactericidal in combination with bactericidal. The regimen consisted of nonsteroidal anti-inflammatory drug (NSAID) and antibiotics. Flunixin meglumine (Loxin, Selmore Pharmaceutical, Pakistan) was used at a dose rate of 2.2 mg/kg (single in a day)

#### 4.5.2. Inclusion Criteria for Animals for Field Trials

- Cattle suffering from clinical mastitis
- Cattle positive for *S. aureus*

*Indicators of Success of Treatment*. The success of treatment was measured based on the absence of clinical signs and clearance of *S. aureus* infection from milk. The latter was done based on bacteriological examination of milk samples as per standard protocols described in Bergey's manual of determinative bacteriology for the identification of bacteria. The presence of any or both indicators were considered a unsuccessful treatment.

### 4.6. Statistical Analysis

A nonparametric test was applied to calculate prevalence and antibiotic susceptibility using SPSS 22 version of statistical computer software. A phylogenetic tree was constructed using Mega X. Nucleic acid and protein motifs were created using MEME Suit (Multiple Expectation maximizations for Motif Elicitation).

Formulae:

(1) $$\begin{array}{c} \text{Prevalence of }S.aureus=\left(\frac{\text{number of }S.aureus\text{ isolated from milk}}{\text{number of milk samples tested}}\right)100,\\ \%\text{susceptibility of }S.aureus\text{ against antibiotics}=\left(\frac{\text{number of }S.aureus\text{ susceptible against antibiotic}}{\text{number of }S.aureus\text{ tested}}\right)100. \end{array}$$

NB: susceptible isolates were either resistant, intermediate, or sensitive which were decided based on their response to antibiotics against set standards.

## 5. Conclusions

Semi-intensive dairy systems were prevalent with antibiotic resistant *S. aureus*. SNPs and change of amino acids in *thermonuclease* protein in *S. aureus* reflected evidence of host shift. On the basis of group of antibiotics, penicillin and glycopeptides were the least effective while macrolides were found the highest efficacious group in an *in-vitro* trial. On an individual antibiotic basis, ampicillin and vancomycin were least effective while enoxacin and sulfamethoxazole/trimethoprim were most effective in an *in-vitro* trial. Response of a single antibiotic regimen, in field trial, supported oxytetracycline while a double antibiotic regimen supported gentamicin with oxytetracycline, cefotaxime with vancomycin, and ciprofloxacin with vancomycin. The study thus proposed adoption of evidence based therapeutics against bacterial pathogens keeping molecular study as an integral part of any treatment protocol.

## Figures and Tables

**Figure 1:** PCR amplicons of nuc gene (*S. aureus*). *M* = 1 kb DNA ladder (gene on 1 kb DNA ladder); Lane 1: Staph-1; Lane 2: Staph-2; Lane 3: Staph-3.

**Figure 2:** Alignment of *S. aureus* nuc gene (Staph-1, Staph-2, Staph-3, and reference).

**Figure 3:** Alignment of *S. aureus* nuc protein (Staph-1, Staph-2, Staph-3, and reference sequence).

**Figure 4:** Nucleotide motifs of *S. aureus* nuc gene.

**Figure 5:** nuc protein motifs of *S. aureus*.

**Figure 6:** Phylogenetic tree of *S. aureus* nuc gene.

**Figure 7:** Gene structure (exonic region) of *S. aureus nuc gene*.

**Figure 8:** Protein structure (exonic region) of *S. aureus* nuc protein.

**Figure 9:** Protein-protein interaction of *S. aureus* nuc protein (Staph-1 protein, Staph-2 protein, and Staph-3 protein).

**Figure 10:** Predicted functional partners of *S. aureus* nuc protein (Staph-1 protein, Staph-2 protein, and Staph-3 protein).

**Figure 11:** Coexpression of *S. aureus* nuc protein (Staph-1 protein, Staph-2 protein, and Staph-3 protein).

**Figure 12:** Distribution of *S. aureus* at different dairy farms; red color indicates positive cases. Percentage is also given in pie chart indicating the percentage of *S. aureus* at different farms which are indicated in different colors.

**Figure 13:** Comparison of percentage susceptibility (resistant, intermediate, and sensitive) isolates of *S. aureus* against individual antibiotics of different classes: (a) penicillin; (b) cephalosporins; (c) aminoglycosides; (d) sulfonamides; (e) macrolides; (f) tetracyclines.

**Figure 14:** Clinical mastitis cases as an indication of inclusion criteria of animals for field trial of antibiotics: (a) udder inflammation, arrow is pointing out; (b) flakes in milk; (c) *S. aureus* growth on mannitol salt agar, arrow pointing out typical pinpoint colonies.

**Table 1:** *S. aureus nuc* protein conserved domain structure (reference sequence, Staph-1, Staph-2, and Staph-3).

Sample ID	Identified domain	Similarity score	Total nr sequences	Total architecture	Conserved domain structure
Reference protein, Staph-1, Staph-2, and Staph-3	Chain A, *staphylococcal* nuclease	1	5902	144	
Staph-1 protein	Chain A, *staphylococcal* nuclease	1	5902	144	
Staph-2 protein	Chain A, *staphylococcal* nuclease	1	5902	144	
Staph-3 protein	Chain A, *staphylococcal* nuclease	1	5902	144	

**Table 2:** *S. aureus nuc* protein physical and chemical properties (Staph-1, Staph-2, Staph-3, and reference sequence).

Sample ID	Reference protein	Staph-1 protein	Staph-2 protein	Staph-3 protein
Number of amino acids	152	152	152	152
MW	16561.02	16637.12	16562.01	16562.01
pI	9.32	9.30	9.2	9.2
Number of negatively charged residues	17	17	18	18
Number of positively charged residues	23	23	23	23
Formula	C_732_H_1194_N_198_O_227_S_5_	C_738_H_1198_N_198_O_227_S_5_	C_732_H_1193_N_197_O_228_S_5_	C_732_H_1193_N_197_O_228_S_5_
Total number of atoms	2356	2366	2355	2355
II	30.78	28.46	30.22	30.22
Aliphatic index	80.79	80.79	80.79	80.79
GRAVY	-0.388	-0.391	-0.388	-0.388

**Table 3:** Average percentages of antibiogram by different classes of antibiogram against *S. aureus*.

Class of antibiotic	Resistant (%)	Intermediate (%)	Sensitive (%)
Penicillins	46.67	26.67	26.66
Cephalosporins	36.67	30	33.33
Aminoglycosides	20	26.67	53.33
Sulfonamides	20	33.33	46.67
Macrolides	33.33	16.67	50
Tetracyclines	23.33	30	46.67
Fluoroquinolones	10	10	80
Glycopeptides	43.33	26.67	30

**(a):** 

Class of antibiotic	Bacteriostatic with bacteriostatic (*n* = 5)				
	Antibiotic with dose rate	Alone	Sulfadimidine	Azithromycin	Oxytetracycline
Aminoglycoside	Gentamicin (G) (2.2-6 mg/kg BW)	2/5 (40%)	3/5 (60%)	2/5 (40%)	4/5 (80%)
Sulfonamide	Sulfadimidine (45 mg/kg BW) IM	2/5 (40%)	—	2/5 (40%)	3/5 (60%)
Macrolide	Azithromycin (A) (6-10 mg/kg BW)	1/5 (20%)	—	—	3/5 (60%)
Tetracycline	Oxytetracycline (O) (17 mg/kg BW)	4/5 (80%)	—	—	—

**(b):** 

Class of antibiotic	Bactericidal with bactericidal (*n* = 5)			
	Antibiotic with dose rate	Alone	Ciprofloxacin	Vancomycin
Cephalosporin	Cefotaxime (Ce) (10 mg/kg BW)	3/5 (60%)	3/5 (60%)	4/5 (80%)
Fluoroquinolones	Ciprofloxacin (Ci) (5-10 mg/kg body weight) (IV)	3/5 (60%)	—	4/5 (80%)
Glycopeptides	Vancomycin (V) (8-12 mg/kg BW) (IV)	3/5 (60%)	—	—

**Table 5:** Names of antibiotics along with their classes used in the study.

Antibiotic group	Name of antibiotic	Antibiotic group	Name of antibiotic
(1) Penicillin	Ampicillin	(2) Macrolides	Erythromycin
	Oxacillin		Azithromycin
	Amoxicillin		Clarithromycin
(3) Cephalosporin	Cefoxitin	(4) Tetracyclines	Tetracycline
	Cefixime		Oxytetracycline
	Cefotaxime		Doxycycline
(5) Aminoglycoside	Streptomycin	(6) Fluoroquinolones	Ciprofloxacin
	Amikacin		Levofloxacin
	Gentamicin		Enoxacin
(7) Sulfonamide	Sulfamethoxazole/trimethoprim	(8) Glycopeptides	Vancomycin
	Sulfaphenazole		Dalbavancin
	Sulfadiazine		Telavancin

## Data Availability

No data were used.

## References

[1] Ramírez-Rivera E. J., Rodríguez-Miranda J., Huerta-Mora I. R., Cárdenas-Cágal A., Juárez-Barrientos J. M. (2019). Tropical milk production systems and milk quality: a review. *Tropical Animal Health and Production*.

[2] Cuny C., Friedrich A., Kozytska S. (2010). Emergence of methicillin-resistant *Staphylococcus aureus* (MRSA) in different animal species. *International Journal of Medical Microbiology*.

[3] Morris W. (2012). *The Collected Works of William Morris: With Introductions by His Daughter May Morris*.

[4] Johnson T. J., Nolan L. K. (2009). Pathogenomics of the virulence plasmids of Escherichia coli. *Microbiology and Molecular Biology Reviews*.

[5] Vanderhaeghen W., Cerpentier T., Adriaensen C., Vicca J., Hermans K., Butaye P. (2010). Methicillin-resistant *Staphylococcus aureus* (MRSA) ST398 associated with clinical and subclinical mastitis in Belgian cows. *Veterinary Microbiology*.

[6] Cosandey A., Boss R., Luini M. (2016). *Staphylococcus aureus* genotype B and other genotypes isolated from cow milk in European countries. *Journal of Dairy Science*.

[7] Reshi A. A., Husain I., Bhat S. A. (2015). Bovine mastitis as an evolving disease and its impact on the dairy industry. *International Journal of Current Research and Review*.

[8] Wells S. J., Ott S. L., Seitzinger A. H. (1998). Key health issues for dairy cattle--new and old. *Journal of Dairy Science*.

[9] Guo Y., Qiu P., Su H. (2021). Antimicrobial resistance and virulence genes distribution in Trueperella pyogenes isolated from dairy cows with clinical mastitis in Liaoning of China. *Pakistan Veterinary Journal*.

[10] Abdeen E. E., Mousa W. S., Abdel-Tawab A. A., El-Faramawy R., Abo-Shama U. H. (2021). Phenotypic, genotypic and antibiogram among *Staphylococcus aureus* isolated from bovine subclinical mastitis. *Pakistan Veterinary Journal*.

[11] Fagundes H., Oliveira C. A. F. (2004). Infecções intramamárias causadas por Staphylococcus aureus e suas implicações em paúde pública. *Ciência rural*.

[12] Iqbal Z., Seleem M. N., Hussain H. I., Huang L., Hao H., Yuan Z. (2016). Comparative virulence studies and transcriptome analysis of *Staphylococcus aureus* strains isolated from animals. *Scientific Reports*.

[13] Altaf M., Ijaz M., Iqbal M. K. (2019). Molecular characterization of methicillin resistant *Staphylococcus aureus* (MRSA) and associated risk factors with the occurrence of goat mastitis. *Pakistan Veterinary Journal*.

[14] Javed M. U., Ijaz M., Fatima Z. (2021). Frequency and antimicrobial susceptibility of methicillin and vancomycin-resistant *Staphylococcus aureus* from bovine milk. *Veterinary Journal*.

[15] Bronner S., Monteil H., Prévost G. (2004). Regulation of virulence determinants in *Staphylococcus aureus*: complexity and applications. *FEMS Microbiology Reviews*.

[16] Cheung A. L., Bayer A. S., Zhang G., Gresham H., Xiong Y. Q. (2004). Regulation of virulence determinants in vitro and in vivo in *Staphylococcus aureus*. *FEMS Immunology and Medical Microbiology*.

[17] Pragman A. A., Schlievert P. M. (2004). Virulence regulation in *Staphylococcus aureus*: the need for in vivo analysis of virulence factor regulation. *FEMS Immunology and Medical Microbiology*.

[18] Dinges M. M., Orwin P. M., Schlievert P. M. (2000). Exotoxins of *Staphylococcus aureus*. *Clinical Microbiology Reviews*.

[19] Tang J., Zhou R., Shi X., Kang M., Wang H., Chen H. (2008). Two thermostable nucleases coexisted in *Staphylococcus aureus*: evidence from mutagenesis andin vitroexpression. *FEMS Microbiology Letters*.

[20] Fang H., Hedin G. (2003). Rapid screening and identification of methicillin-resistantStaphylococcus aureusfrom clinical samples by selective-broth and real-time PCR assay. *Journal of Clinical Microbiology*.

[21] Akkou M., Bouchiat C., Antri K. (2018). New host shift from human to cows within *Staphylococcus aureus* involved in bovine mastitis and nasal carriage of animal's caretakers. *Veterinary Microbiology*.

[22] Knight G. M., Budd E. L., Whitney L. (2012). Shift in dominant hospital-associated methicillin-resistant *Staphylococcus aureus* (HA-MRSA) clones over time. *Journal of Antimicrobial Chemotherapy*.

[23] Vincze S., Stamm I., Kopp P. A. (2014). Alarming proportions of methicillin-resistant *Staphylococcus aureus* (MRSA) in wound samples from companion animals, Germany 2010-2012. *PLoS One*.

[24] Franck K. T., Gumpert H., Olesen B. (2017). Staphylococcal aureus enterotoxin C and enterotoxin-like L associated with post-partum mastitis. *Frontiers in Microbiology*.

[25] O’Dea M., Abraham R. J., Sahibzada S. (2020). Antimicrobial resistance and genomic insights into bovine mastitis-associated *Staphylococcus aureus* in Australia. *Veterinary Microbiology*.

[26] Fursova K., Sorokin A., Sokolov S. (2020). Virulence factors and phylogeny of *Staphylococcus aureus* associated with bovine mastitis in Russia based on genome sequences. *Science*.

[27] Moretti R., Soglia D., Chessa S. (2021). Identification of Snps associated with somatic cell score in candidate genes in Italian Holstein Friesian bulls. *Animals*.

[28] Ali A. O., Mahmoud H. Y. (2016). Sequencing and phylogenetic characterization of *S. aureus* thermonuclease gene. *Assiut Veterinary Medical Journal*.

[29] Kwok A. Y. C., Chow A. W. (2003). Phylogenetic study of Staphylococcus and Macrococcus species based on partial Hsp 60 gene sequences. *International Journal of Systematic and Evolutionary Microbiology*.

[30] Yang W.-T., Ke C.-Y., Wu W.-T., Lee R.-P., Tseng Y.-H. (2019). Effective treatment of bovine mastitis with intramammary infusion of Angelica dahurica and Rheum officinale extracts. *Evidence-based Complementary and Alternative Medicine*.

[31] Sasaki T., Kikuchi K., Tanaka Y., Takahashi N., Kamata S., Hiramatsu K. (2007). Reclassification of phenotypically identified Staphylococcus intermedius strains. *Journal of Clinical Microbiology*.

[32] Ciftci A., Findik A., Onuk E. E., Savasan S. (2009). Detection of methicillin resistance and slime factor production of *Staphylococcus aureus* in bovine mastitis. *Brazilian Journal of Microbiology*.

[33] Hida Y., Uemura K., Sugimoto H. (2019). Evaluation of performance of the GENECUBE assay for rapid molecular identification of *Staphylococcus aureus* and methicillin resistance in positive blood culture medium. *PLoS One*.

[34] Hegde R., Isloor S., Prabhu K. N. (2013). Incidence of subclinical mastitis and prevalence of major mastitis pathogens in organized farms and unorganized sectors. *Indian Journal of Microbiology*.

[35] Lodhi F. L., Saleem M. I., Aqib A. I. (2021). Bringing resistance modulation to epidemic methicillin resistant *S. aureus* of dairy through antibiotics coupled metallic oxide nanoparticles. *Microbial Pathogenesis*.

[36] Naseer M. A., Aqib A. I., Ashar A. (2021). Detection of altered pattern of antibiogram and biofilm character in *Staphylococcus aureus* isolated from dairy milk. *Pakistan Journal of Zoology*.

[37] Shoaib M., Rahman S. U., Aqib A. I. (2020). Diversified epidemiological pattern and antibiogram of MecA gene in *Staphylococcus aureus* isolates of pets, pet owners and environment. *Pakistan Veterinary Journal*.

[38] Sarwar I., Ashar A., Mahfooz A. (2021). Evaluation of antibacterial potential of raw turmeric, nano-turmeric, and NSAIDs against multiple drug resistant *Staphylococcus aureus* and E. coli isolated from animal wounds. *Pakistan Veterinary Journal*.

[39] Aqib A. I., Ijaz M., Anjum A. A. (2017). Antibiotic susceptibilities and prevalence of methicillin resistant *Staphylococcus aureus* (MRSA) isolated from bovine milk in Pakistan. *Acta Tropica*.

[40] Shafique L., Wu S., Aqib A. I. (2021). Evidence-based tracking of MDR E. coli from bovine endometritis and its elimination by effective novel therapeutics. *Antibiotics*.

[41] Su Y., Yu C.-Y., Tsai Y., Wang S.-H., Lee C., Chu C. (2016). Fluoroquinolone-resistant and extended-spectrum *β*-lactamase-producing _Escherichia coli_ from the milk of cows with clinical mastitis in Southern Taiwan. *Journal of Microbiology, Immunology and Infection*.

[42] Clinical and Laboratory Standards Institute (2019). Clinical and Laboratory Standards Institute.

[43] The European Committee on Antimicrobial Susceptibility Testing (2020). EUCAST disk diffusion test manual. Version 8.0. http://wwweucastorg/.

[44] Bondoc I., Șindilar E. V. (2002). *Veterinary sanitary control of food quality and hygiene (Controlulsanitarveterinar al calitățiișisalubritățiialimentelor – original title). Vol. I*.

[45] Bondoc I. (2007). *Technology and quality control of milk and dairy products (Tehnologiașicontrolulcalitățiilapteluișiproduselor lactate – original title). Vol. I*.

